# Design, Synthesis, and Quorum Quenching Potential of Novel Catechol–Zingerone Conjugate to Find an Elixir to Tackle *Pseudomonas aeruginosa* Through the Trojan Horse Strategy

This article has been retracted.

**DOI:** 10.3389/fchem.2022.902719

**Published:** 2022-06-15

**Authors:** Surabhi Mangal, Tamanna Dua, Monika Chauhan, Neelima Dhingra, Sanjay Chhibber, Vasundhara Singh, Kusum Harjai

**Affiliations:** ^1^ Department of Microbiology, Panjab University, Chandigarh, India; ^2^ Department of Applied Sciences, Punjab Engineering College (Deemed to be University), Chandigarh, India; ^3^ University Institute of Pharmaceutical Sciences (UIPS), Panjab University, Chandigarh, India

**Keywords:** *Pseudomonas aeruginosa*, catechol, xenosiderophore, Trojan horse strategy, multidrug resistance, zingerone

## Abstract

To address the issue of multidrug resistance in *Pseudomonas aeruginosa*, a novel catechol–zingerone conjugate (**1**) linked *via* a non-hydrolyzable 1,2,3-triazole linker was synthesized and subjected to biological evaluation based on the Trojan horse strategy. To enhance the efficacy, catechol, a xenosiderophore, utilized by *P. aeruginosa* for iron assimilation, and the dietary phytochemical zingerone, known for its anti-virulent activity against *Pseudomonas aeruginosa*, were exploited in the present study. Theoretical validation of conjugate (**1**) was conducted by *in silico* molecular docking analysis to determine the interaction with outer membrane transport receptor PirA and quorum sensing signal receptors. In addition, nine-fold binding affinity of Conjugate (**1**) toward PirA (5FP2) in comparison to its natural ligand catechol with D-score −1.13 Å authenticated the designed Trojan horse drug. Conjugate (**1**) showed stronger anti-virulent activity than zingerone; hence, it exhibited a promising anti-biofilm efficacy as assessed by crystal violet assay and visualized by FESEM toward *P. aeruginosa*. Encouraging results against *P. aeruginosa* in terms of quorum sensing regulated virulence factors, motility phenotypes, and biofilm formation with no cell cytotoxicity and could help open hitherto unexplored possibilities of establishing Trojan horse drugs as a successful approach against multidrug resistance in *P. aeruginosa*.

## 1 Introduction

Antimicrobial resistance constitutes one of the paramount issues threatening global health. *Pseudomonas aeruginosa*, one of the Gram-negative ESKAPE pathogen, is responsible for 10% of the hospital-acquired infections, including chronic cystic fibrosis (Lyczak et al., 2000; Rao et al., 2011). This high-priority pathogen could forgo the effect of the approved families of antibiotics through several mechanisms mainly by alteration of target protein, increased efflux, restricted antibiotic penetration, and enzymatic degradation of drug (Gao et al., 2018; Gatadi et al., 2019). New strategies to bypass resistance mechanisms are urgently needed (Chellat et al., 2016; Gonzalez-Bello, 2017; WHO, 2017). One such approach is the Trojan horse strategy which can specifically deliver the drugs through outer membrane receptors (Tilloston, 2016; Klahn and Bronstrup, 2017).

In view of the fact that bacteria need micromolar concentration of iron to facilitate its growth and virulence, bacteria can acquire iron by producing their own siderophores through active transport processes (Hider and Kong, 2010). Most of them belong to one of the four groups, depending on the structure of the iron-chelating fragment of the siderophore: 1) catecholates, 2) hydroxamic acids, 3) α-hydroxycarboxylic acids, and 4) mixed-type. *P. aeruginosa* produces two major siderophores, pyoverdin and pyochelin. Many studies have shown that siderophore iron uptake pathways can be used to transport antibiotics into bacteria (Mollmann et al., 2009; Ji et al., 2012). Such an approach has already been developed with pyoverdin, the primary siderophore of *P. aeruginosa* mediating the iron uptake system, and some siderophore drug conjugates based on pyoverdin have already been reported (Mislin and Schalk, 2014). Pyoverdine–ampicillin conjugate displays potent antibacterial activity against the producer strains of *P. aeruginosa*, while the bacteria were resistant to ampicillin alone (Kinzel et al., 1998). A disadvantage of the pyoverdine iron uptake system is that each strain of *P. aeruginosa* produces its own pyoverdine along with a corresponding species transporter. On the other hand, pyochelin (Pch), the second-most common siderophore of *P. aeruginosa*, is reported to be conserved and produced by all the strains of *P. aeruginosa* and *Burkholderia cepacia.* Modified pyochelin was utilized for the construction of pyochelin–fluoroquinolone conjugates bearing a cleavable linker (Rivault et al., 2007). Few pyochelin–antibiotic conjugates have also been synthesized, showing negligible or weak antimicrobial activity (Mislin and Schalk, 2014).

There are several inherent problems which need to be addressed before the development of a hybrid drug especially if the agent is directed at Gram-negative pathogens. Limited cellular penetration across the dual layer of Gram-negative bacteria is the first major concern for hybrid agents that have molecular mass of > 600 g/mol. Using catechol, a siderophore entity, as a starting point for drug conjugate may enable solving the problem of penetration and may also enhance the permeability by exploiting the iron uptake system. Studies have reported that siderophore components in conjugates do not necessarily have to identically replicate the natural siderophores (Lin et al., 2019). Also, *P. aeruginosa* can acquire iron through siderophores from other microorganisms called xenosiderophores or siderophore piracy. Therefore catechol, having a simplified structure with no bulky side groups, can be exploited as a carrier for drug penetration, using bacterial iron uptake systems (Cir and Fiu in *E. coli* and PfeA and PirA in *P. aeruginosa*), having less chances of steric hindrance during conjugation.

The other problem lies within the fundamental idea of covalently linking two entities together. The point of attachment and physicochemical properties of the chosen linker are crucial for the overall activity of the hybrid. The linker group connects the vector with the drug and hence acts as a key component in the function and effectiveness of the conjugate. Linkers can be cleavable either by enzyme catalysis or by hydrolysis and non-cleavable which are stable to metabolic degradation. The prerequisite attributes of an ideal linker includes less toxicity, high stability in the biological system, and specific release of the drug. Triazole, being stable to metabolic degradation along with its improved solubility due to formation of hydrogen bonding, can be used as a non-cleavable linker.

The trend of using natural products for treating diseases is increasing due to persisting drug resistance. Zingerone (4-para methoxy-4-hydrophenyl-2 butanone, vinillyl acetone) is mainly found in dry ginger root and also produced by gingerols and shogoals. The retro-aldol reaction results in the conversion of gingerol (component of ginger) into zingerone on cooking. It has been observed in our previous research that zingerone attenuates cell surface properties, making *P. aeruginosa* highly susceptible for killing with antibiotics and by serum and phagocytes, components of innate immunity (Kumar et al., 2015). Studies have shown the protective effect of zingerone against radiation-induced DNA damage and antiapoptotic effect in human lymphocytes (Rao et al., 2011). Therefore, we selected zingerone as a drug to be delivered using the Trojan horse strategy using the catechol-mediated iron acquisition pathway.

With the aim of developing more potent and better targeted drugs by following the Trojan horse strategy, the present study is designed to synthesize a hybrid drug, catechol–zingerone, to be used against *P. aeruginosa.* Past studies have demonstrated the presence of catecholate-binding outer membrane proteins (e.g., PirA) and the quorum sensing signal receptor proteins (e.g., LasR, RhlR, PqsR, and TraR) in *P. aeruginosa* (Moynie et al., 2019; Bose et al., 2020). In order to validate the hypothesis of this conjugated system as a potential quorum quenching agent, a molecular docking approach was utilized to understand the putative binding affinities of the catechol–zingerone conjugate (1) toward surface receptor and quorum sensing proteins, followed by *in vitro* and *ex vivo* studies. This approach will not only help in disarming the pathogen of its virulence, making it susceptible to host defenses, but also will alter the minimum inhibitory concentration (MIC) of antibiotics, hence overcoming the menace of development of antibiotic resistance.

## 2 Materials and Methods

### 2.1 Molecular Docking

#### 2.1.1 Target Identification

The 3D crystallographic structure for Pir A (PDB: 5FP2), LasR (PDB: 2UV0), PqsR (4JVI), TraR (1HOM), and RhlR HM (P54292) was retrieved from a protein data bank http://www.rcsb.org. For RhlR, the targeted amino acid sequence P54292 was obtained from the UniProt KB database (http://www.uniprot.org/) to perform homology modeling.

#### 2.1.2 Protein Preparation

To prepare the target protein, the protein structure was analyzed, reprocessed, and refined using the protein preparation protocol. The protocol was performed by removal of water molecules and protonation of titratable residues to stabilize the receptor protein. Furthermore, protein structure integrity was assessed and checked for its missing residues, followed by insertion of loop regions and missing atoms near the active site, using a loop builder tool. Furthermore, co-factors and external ligands present in the crystal structure were deleted and extracted out. Ultimately, final protein was saved in .mol format as a receptor. At the same time, homology modeling was performed for the RhlR selecting a suitable template for each target sequence using the BLAST tool.

#### 2.1.3 Ligand Standardization

One of the important determinants for a successful docking is the structure of the ligand. The ChemDraw ultra 12.0 software was used to draw the structure of catechol–zingerone conjugate (**1**) and natural ligands (catechol, 3-oxo-C12-HSL, PQS, 3-oxo-C8-HSL, and C4-HSL). However, energy calculation and optimization of structural geometry were performed using VLife MDS 4.6 software. The two-dimensional (2D) structures were transformed into three-dimensional (3D) structures by using the converter module of the VLife module. The 3D structures were then subjected to energy minimization and geometry optimization using the Merck Molecular Force Field (MMFF) method. Conformers with lowest energy were selected for docking simulation studies. The comprehensive and integrated graphical user interface program of the Vlife MDS 4.6, that is, “Bio Predicta module” was used to prepare, run, and analyze the docking simulations on the HP Pentium IV 2.80 GHz Processor/Microsoft Win XP Home Edition system.

### 2.2 General Methods for Chemistry

All reagents and solvents were purchased from Merck and Aldrich companies without any purification. The reaction progress and the purity of synthesized compounds were monitored by thin-layer chromatography (TLC) using silica gel plates with Fluorescence F254 and UV visualization. Flash chromatography was performed by using a 230–400 mesh silica gel and the indicated solvent system. ^1^H NMR spectra were recorded on a Bruker AV-400 spectrophotometer at 400 MHz or a Bruker AV-500 spectrophotometer at 500 MHz. ^13^C NMR spectra were recorded on a Bruker AV-500 spectrophotometer at 125 MHz. Coupling constants (*J*) are expressed in hertz (Hz). Chemical shifts were reported in parts per million (ppm) relative to an internal standard (tetramethylsilane). Proton coupling patterns were described as singlet (s), doublet (d), triplet (t), quartet (q), multiplet (m), and broad (b). Mass spectra were recorded on an LCMS-Q-TOF (Waters) by means of the ESI method. The elemental analysis for C, H, and N was carried out with an elemental analyzer GmbH VarioEL. Purity of the compound was determined by reverse-phase high-performance liquid chromatography [HPLC, Waters (Column: Waters C18, 5.0 µm, 4.6 × 250 mm) detection wavelength 210 nm; temperature 60°C] to be >95%. A flow rate of 1.0 ml/min was used with the mobile phase of acetonitrile in water with 0.1% modifier (orthophosphoric acid. v/v).

#### 2.2.1 Synthesis of Compound **4**

To a stirred solution of 1-azido propylamine **3** (240 mg) in anhydrous CH_2_Cl_2_ (5 ml) at 20°C was dropwise added a solution of pentafluorophenyl ester **2** (1.0 g) in a minimum volume of anhydrous CH_2_Cl_2_ (5 ml). The resulting mixture was stirred at 20°C for 3 h and TLC-monitored. On completion of the reaction, the solvent was evaporated under reduced pressure. The crude mixture was purified on a silica gel column (hexane: ethyl acetate 8:2) to afford compound **4** in the form of yellow oil in 80% yield (m.p.: 148°C).

^1^H NMR (500 MHz, CDCl_3_): 7.53–7.58 (m, 5H), 7.40–7.43 (m, 5H), 7.31 (t, *J* = 5.5 Hz, 4.8 Hz, 1H),7.01 (dd*, J* = 1.3 Hz,1H), 6.94 (t, *J* = 8.0 Hz, 1H), 3.60(q,*J* = 6.5 Hz, 2H), 3.44 (t, *J* = 6.5 Hz, 2H), and 1.92 (t, *J* = 6.6 Hz, 2H).

^13^C NMR (100 MHz, DMSO): δ 162.88, 146.75, 144.26, 139.18, 129.39, 128.43, 125.78, 121.81, 121.42, 117.02, 116.83, 111.13, 48.64, 36.67, and 28.32.

MS (ESI): m/z 400.15 [M + H+] HRMS (ESI): C_23_H_20_N_4_O_3_: calcd. 400.44, found 400.55.

IR (KBr, cm^−1^): 3,426, 2,921, 2,100, 1,648, 1,593, 1,536, 1,501, 1,456, 1,250, 1,210, 1,052, 1,019, 747, and 700.

#### 2.2.2 Synthesis of 3-Methoxy-4-(2-Propyne-1-Yloxy)-Phenyl-2-Butanone (**6**)

To a stirred solution of zingerone (1 g, 5.1 mmol) in dry acetone (20 ml), K_2_CO_3_ (1.06 g) and propargyl bromide (0.5 ml, 4.9 mmol) were added dropwise. The mixture was stirred at 60°C for 24 h and quenched with H_2_O at 0°C. Acetone was removed under reduced pressure, and the product was extracted with CH_2_Cl_2_. The organic layer was washed with saturated NaHCO_3_ and brine, dried over MgSO_4_, filtered, and concentrated. The product was obtained as brown solid (1.1 g) in quantitative yield (1.1 g). (m.p.: 197°C).

^1^H NMR (500 MHz, CDCl_3_): δ 6.94(d, *J* = 8.1 Hz 1H), 6.73 (d, *J* = 1.9 Hz, 1H), 6.71 (dd, *J* = 2.0 Hz, 1H), 4.72 (d, *J* = 2.4 Hz, 2H), 3.86 (s, 3H), 2.84(t, *J* = 7.3 Hz, J = 7.6 Hz, 2H), 2.74 (t, *J* = 7.7 Hz, 2H), 2.49 (t, *J* = 2.4 Hz, 1H), and 2.13 (s, 3H).

^13^C NMR (125 MHz, DMSO): δ 207.64, 149.05, 144.53, 134.85, 119.62, 114.39, 112.40, 79.43, 77.92, 56.07, 55.33, 44.23, 29.61, and 28.63.

MS (ESI): m/z 218.25 [M + H+] HRMS (ESI): C_13_H_14_O_3_: calcd. 218.25, found 218.

IR (KBr, cm^−1^): 3,434, 3,248, 2,915, 2,125, 1,706, 1,589, 1,513, 1,450, 1,423, 1,370, 1,329, 1,249, 1,160, 1,134, 1,021, 802, 715, 621, 543, and 447.

#### 2.2.3 Synthesis of Conjugate **1**

To a solution of azido-catechol **4** (112 mg, 1.1 eq.) and alkyne **6** (60 mg, 1 eq.) in THF (1 ml per 0.1 mmol) was added successfully 0.8 M aqueous solution of copper sulfate (1 eq.) and sodium ascorbate (4.7 eq.). The suspension was sonicated and stirred under argon at room temperature (21–23°C). The reaction mixture was filtered on a celite pad and purified on a silica gel column (CH_2_Cl_2_: MeOH) to afford the expected conjugate. For the release of the catechol moiety, conjugates were dissolved in methanolic HCl (6 ml) and further stirred overnight before being evaporated under reduced pressure. The residue was suspended in a minimum of THF, and cyclohexane was added until precipitation of expected conjugate (103 mg) in 60% yield. (m.p.: 248°C).

^1^H NMR (500 MHz, DMSO): δ 12.68 (s, 1H), 9.13 (s, 1H), 8.83 (t, *J* = 5.4 Hz, 5.5 Hz, 1H), 8.23 (s, 1H), 7.27 (dd, *J* = 1.2 Hz, 1H),6.99 (d, *J* = 8.2 Hz, 1H), 6.92 (dd, *J* = 1.2 Hz, 1H), 6.83 (d, *J* = 1.9 Hz, 1H), 6.68–6.71 (m, 2H), 5.05 (s, 1H), 4.44 (t, *J* = 7 Hz, 2H), 3.73 (s, 3H), 3.30–3.33 (m, 2H), 2.69–2.75 (m, 4H), 2.10–2.15 (m, 2H), and 2.09 (s, 3H).

^13^C NMR (125 MHz, DMSO): δ 207.67, 169.86, 149.53, 148.91, 146.11, 145.54, 142.73, 134.27, 124.50, 119.75, 118.72, 117.79, 117.05, 114.82, 113.89, 112.35, 61.84, 55.29, 47.23, 44.28, 36.25, 30.56, 29.62, and 28.65.

MS (ESI): m/z 468.20 [M + H+]. HRMS (ESI): C_24_H_28_N_4_O_6_: calcd. 468.20, found 469.3.

IR (KBr, cm^−1^); 3,386, 2,928, 1,710, 1,641, 1,594, 1,545, 1,513, 1,459, 1,328, 1,262, 1,228, 1,158, 1,139, 1,010, 1,031, 835, 802, 742, 630, 591, and 546.

CHN: C = 60.52, H = 6.23, and N = 11.07

HPLC analysis: ACN:H_2_O (65:35), 12.53 min, 95.5% purity.

### 2.3 Bacterial Strains and Growth Conditions

A standard strain of *P. aeruginosa* PAO1(MTCC-3541) was obtained from Dr. Barbara H. Iglweski, Department of Microbiology and Immunology, University of Rochester, New York (United States). *Agrobacterium tumefaciens* A136 was obtained from J. Handlesman, Wisconsin University (WI, United States) and was used as a biosensor strain. All the strains were maintained in glycerol (50%) and stored at −80°C. Fresh stocks were subcultured for every new experiment. Working solutions of compounds were prepared in 5% (v/v) DMSO supplemented with 0.01% Tween 80.

### 2.4 CAS Assay

To check the iron chelation activity of the synthetic catechol–zingerone conjugate, the CAS agar plates were prepared (Schwyn and Neilands, 1987). Wells (∼9 mm) were cut in the agar plates. The stock solution of 50 µM of synthetic catechol–zingerone conjugate **1**, Compound **6**, zingerone **5**, and 10% DMSO was added into the wells. Color change was observed after 12 h at room temperature.

### 2.5 Antibacterial Activity

To assess the antimicrobial activity against *P. aeruginosa*, a standard agar disc-diffusion method based on the document M2-A8 of CLSI (2003a) was used, whereby the diameters of zones of inhibition around the wells with the test compounds on the surface of *P. aeruginosa* were measured.

### 2.6 AHL Extraction and Anti–Quorum Sensing Activity of the Compounds

AHLs were extracted using the method of Gupta et al., 2011a. Briefly, *Pseudomonas aeruginosa* PAO1 was grown overnight in Luria Broth (14-16h) and was centrifuged at 4°C for 10° min at 3,000 ×g to obtain the cell-free supernatant. AHLs were extracted from the supernatant using an equal volume of acidified ethyl acetate (0.01% acetic acid) and was kept overnight at 4°C. An organic layer was separated and concentrated under reduced pressure. The QS inhibition effect (QSI) was determined by performing the qualitative assay using *A. tumefaciens* A136 (Vattem et al., 2007). In the presence of AHLs, LacI:Z genes get activated and transcripts the reporter gene for the production of blue color in the presence of X-Gal. A Luria agar plate was spread with X-Gal (5-bromo-4-chloro-3-indolyl-β-D-galactopyranoside) and extracted AHLs and *A. tumefaciens* A136 after respective intervals. Conjugate **1**, compound **6**, and zingerone at a concentration of 50 µM were added in wells, and plates were incubated at 30°C. Diameters of the zone of turbidity were measured to assess the QSI activity of the agent.

### 2.7 Estimation of Virulence Factors

Virulence factors were estimated in the cell-free supernatant of *P. aeruginosa* and grown in presence and absence of compounds, that is, 50 µM of synthetic catechol–zingerone conjugate **1**, compound **6**, and zingerone **5**.

#### 2.7.1 Pyocyanin Production

Pyocyanin, a blue green pigment produced by *P. aeruginosa*, was quantified by the method of Huerta et al. (2008). Briefly, 1.5 ml of the chloroform was added to 3 ml of the cell-free supernatant followed by 30 min incubation. Pyocyanin containing a chloroform layer was separated, and absorbance was measured at 690 nm.

#### 2.7.2 Protease Production

Proteolytic activity was quantified in the cell-free supernatant (Visca et al., 1992). In brief, 200 µl of Azocasein (3 mg/ml stock prepared in 0.05 mM Tris-HCl buffer (pH 7.0) supplemented with 0.5 mM CaCl_2_) was added to 200 µl of the cell-free supernatant. After incubation, an equal volume of trichloroacetic acid (TCA) was added to stop the reaction. Absorbance of the supernatant was measured after centrifugation at 420 nm.

#### 2.7.3 Elastase Production

The elastolytic activity was measured using elastin Congo red as the substrate (Visca et al., 1992). Briefly, 1 ml supernatant was mixed with 5 mg of the elastin Congo red in 100 mM Tris-HCl buffer (pH 7.0) and incubated at 37°C for 2 h under shaking conditions. OD was measured after centrifugation at 495 nm.

#### 2.7.4 Alginate Production

Alginate concentration was assessed in the supernatant (Mathee et al., 1999). Briefly, the alginate was precipitated in the supernatant with an equal volume of 2% (w/v) cetylpyridinium chloride followed by centrifugation at 10,000°rpm for 20 °min. The alginate pellet obtained was resuspended in 5 ml of 1 M NaCl and precipitated again with 5 ml of ice-cold 2-propanol. After centrifugation at 10,000 rpm for 10°min, the alginate pellet obtained was resuspended in saline depending on alginate quantity. The carbazole/borate method (Knutson and Jeanes, 1968) was used to quantify alginate. Alginate concentration was determined by measuring OD at 500 nm.

#### 2.7.5 Pyochelin Production

Pyochelin was estimated by using an Arnow assay (Arnow, 1937). A volume of 1°ml of the cell-free supernatant was mixed with 1 ml of nitrite molybdate solution, 1 ml of sodium hydroxide solution (NaOH), and 1 ml of 0.5 N hydrochloric acid (HCl). Final volume makeup was carried out with water, and absorbance was measured at 510 nm.

#### 2.7.6 Hemolysin Production

To quantify the concentration of cell-free hemolysin (CFH) and cell bound-hemolysin (CBH), the cell-free supernatant and cells (10^8^ CFU/ml) were used (Landkish and Vogt, 1972). Briefly, 1.5 ml of 2% sheep RBC suspension was mixed with 1.5 ml of treated and untreated cell-free supernatant as well as cell suspension. After 2°h of the incubation, the tubes were centrifuged at 3,000 °rpm for 15° min. Absorbance was measured at 545 nm.

#### 2.7.7 Cell Surface Hydrophobicity Assay

The method of Rosenberg et al. (1986) was used to measure cell surface hydrophobicity. Planktonic cells (10^8^ cfu/ml) grown in the presence and absence of conjugate **1**, compound **6**, and zingerone alone were harvested, washed, and resuspended in PBS (Ph-7.2). Initial OD _(i)_ was measured at 600 nm. A volume of 0.35 ml of xylene was added, and cells were vortexed for 1 min. After phase separation, final O.D of the aqueous phase was measured at 600 nm and expressed as O.D. _(f)_ Surface hydrophobicity of each strain was expressed as percent hydrophobicity.

$$\%\;\text{Hydrophobicity}=\left[\left({\text{OD}}_{\left(\text{i}\right)}-\text{O}\text{.D}\text{.}(\text{f})/\text{OD}\left(i\right)\right)\times 100\right].$$

### 2.8 Motility Phenotypes

#### 2.8.1 Swarming Motility

To study the effect of conjugate **1**, compound **6**, and zingerone **5** at a concentration of 50 µM on motility phenotypes, the cells of *P. aeruginosa* grown in presence and absence of sub MIC of treatment regime were point-inoculated on swarm agar plates (nutrient broth 0.8%, D-glucose 0.5%, and agarose 0.5%). Swarming motility was determined by measuring turbid circular zones after 24 h of incubation at 37°C.

#### 2.8.2 Swimming Motility

To assess the swimming motility, treated and untreated cells of *P. aeruginosa* were inoculated on swim agar plates (tryptone 1%, Nacl 0.5%, and agarose 0.3%). After 24 h of incubation at 30°C, the plates were observed for the swimming motility around the point inoculation.

#### 2.8.3 Twitching Motility

To assay twitching motility, *P. aeruginosa* cells with and without treatment were stabbed in LB plates (bacto agar 1%). After 24 h of incubation at 37°C, a hazy zone of growth at the interface of the agar was measured.

### 2.9 Anti-Fouling Effect of Catechol–Zingerone Conjugates

#### 2.9.1 Qualitative Biofilm Generation Assay

A volume of 3 ml LB in polypropylene microcentrifuge tubes (Tarson, Kolkata, India) was inoculated with 50 µl of an overnight grown culture (1 × 10^6^ CFU/ml) of *P. aeruginosa.* Conjugate **1**, compound **6**, and zingerone alone were added to tubes at sub-MIC concentration (50 µM). A tube without conjugate **1** served as the control. The tubes were incubated for 24 h. The media containing loose planktonic cells were discarded and washed thrice with phosphate-buffered saline (PBS). After washing, the adherent cells were stained with 0.1% crystal violet (CV). After 30° min, the tubes were washed with distilled water to remove excess stain. The color intensity was examined to assess biofilm formation. Adherence ranged from weak (+) to strong (+++).

#### 2.9.2 Quantitative Biofilm Inhibition Assay

Biofilm inhibition ability of conjugate **1**, compound **6**, and zingerone was studied on polystyrene 96-well microtiter plates (Laxbo Manufacturing Co., Pune, India). Diluted mid-log phase cells of *P. aeruginosa* (1 × 10^6^ CFU/ml) were added to different wells of the microtiter plate and supplemented with sub-MIC concentration, that is, 50°µM of conjugate **1**, compound **6**, and zingerone **5** alone. Bacterial culture without treatment served as the control. The attached biofilm cells were stained with CV after discarding media containing planktonic cells alone with the PBS washings. Absorbance was measured on each day after elution of stain with ethanol. The wells were processed in a similar way up to 7°days.

#### 2.9.3 Preformed Biofilm Eradication Assay

A volume of 100 μl of diluted culture (1 × 10^6^ CFU/ml) was added to wells of the microtiter plate. The preformed peak (4°days old) biofilm was treated with 50 µM of conjugate **1**, compound **6**, and zingerone alone. Untreated wells served as the control. The media containing loose planktonic cells were discarded and washed thrice with phosphate-buffered saline (PBS) followed by staining with CV for 30 min. Stain was eluted with ethanol followed by absorbance at 545 nm.

#### 2.9.4 EPS Production

The interference of conjugate **1**, compound **6**, and zingerone alone on EPS production by the *P. aeruginosa* biofilm was evaluated by using the Congo red binding assay (Goswami et al., 2014). The peak day (4°days old) pre-formed biofilms in the microtiter treated with 50 µM (sub-MIC concentration) of conjugate **1**, compound **6**, and zingerone alone at sub-MIC concentration were incubated for 24 h at 37°C. Planktonic cells were discarded and washed thrice with PBS. Congo red (1%, w/v) was added to each well and incubated in dark for 30° min. Excess dye was removed with distilled water, and the stain was eluted with DMSO. Absorbance was measured at 490 nm in an ELISA reader (REMI).

#### 2.9.5 Microscopic Examination of *Pseudomonas aeruginosa* Biofilms

Microscopic analysis of biofilms was performed by SEM (Hawser and Douglas, 1994). Biofilms of *P. aeruginosa* were formed on sterile conditions on catheter (1 × 1°cm). The biofilms were grown in the absence and presence of conjugate **1**, compound **6**, and zingerone. The peak day biofilms were fixed with 2.5% (v/v) glutaraldehyde in PBS for 1 h at room temperature in dark. After washing, dehydration was performed in ethanol with different concentrations (50%, 60%, 70%, 80%, 90%, and 100%). Catheters were dried, gold-coated, and viewed under a field emission scanning electron microscope (FESEM, SU8010, Hitachi, Tokyo, Japan).

### 2.10 Mechanism of Membrane Disruption

#### 2.10.1 Reduction of Membrane Potential

The influence of conjugate **1**, compound **6**, and zingerone on membrane permeability was detected by using a crystal violet uptake assay (Devi et al., 2010). Suspensions of *P. aeruginosa* (1 × 10^6^ CFU/ml) were prepared in LB broth. The cells were harvested, washed twice, and suspended in 50 mM PBS (pH 7.4). Conjugate 1 at the concentration of 100 µM was added to the cell suspension and incubated at 37°C for 30 min. Suspension without treatment served as the control. The cells were harvested at 10,000 rpm for 5 min and suspended in PBS containing 10 μg/ml of crystal violet. Aliquots of 1 ml were removed at different time intervals (10, 20, 40, and 60 min) and centrifuged at 10,000 rpm for 5°min, after which OD_590_ of the supernatant was measured. The OD value of crystal violet solution, which was originally used in the assay, was considered 100% excluded. The percentage of crystal violet uptake was calculated using the following formula:

% Dye uptake=100−[(OD of the sample/ OD value of crystal violet solution)×100].

#### 2.10.2 Release of Cellular Material

Enumeration of release of cellular materials from *P. aeruginosa* was determined by using the Bradford reagent Devi et al., 2010). Overnight grown cultures (1 × 10^6^ CFU/ml) were harvested at 8,000 rpm, washed twice with NaCl (0.85%), and finally suspended in 1 ml of saline in the presence of treatment regimes and incubated at 37°C. Suspension without treatment served as the control. After the incubation of 60 and 120°min, aliquots of 1 ml were removed and centrifuged at 10,000 rpm for 5 min. Absorbance of the supernatant was then measured at 260 nm. The results were expressed in the form of OD recorded at each time interval. To confirm membrane disintegration of *P. aeruginosa* by the conjugate, released membrane proteins were also detected by SDS-PAGE. Intensities of separated bands increased from 60 to 120 min and showed a distinct banding pattern as compared to the control (untreated).

### 2.11 *Ex-Vivo* Efficacy of Conjugate

#### 2.11.1 Mice and Ethics Statement

Female 6–8°week-old BALB/c mice (weighing 20–30 g), bred and procured from the Central Animal House, Panjab University, Chandigarh, India, were used in the present study. The mice were housed in polypropylene cages and bedded with dry and clean husk with proper ventilation of the room. The animals were fed on standard pellets of antibiotic-free synthetic diet (Hindustan Unilever Ltd., Mumbai, India) and water *ad libitum*. The ethical clearance to conduct the experiment was approved by the Institutional Animal Ethics Committee of Panjab University, Chandigarh, India (Approval No. PU/45/99/CPCSEA/IAEC/2021/491). All the experimental protocols were followed according to the guidelines of the Committee for the Purpose of Control and Supervision of Experiments on Animals (CPCSEA), Government of India.

#### 2.11.2 Cytotoxicity Assay

The conjugate **1**, compound **6**, and zingerone alone were evaluated for cytotoxicity using the 3-(4,5-dimethylthiazol-2-yl)-2,5-diphenyl-2H-tetrazolium bromide (MTT) reduction assay method of Mosmann (1983). Mouse macrophages were seeded (2× 10^5^ cells/ml) in a 96-well plate and cultured overnight to obtain a monolayer. The cells were then treated with conjugate **1**, compound **6**, and zingerone alone at sub-MIC concentration and were incubated at 37°C for 24 h in a CO_2_ incubator. After incubation, the cells were exposed to MTT solution (5 mg/ml) for 4 h at 37°C. Media were removed, and the formed formazan crystal was solubilized with 200 μl of 100% ethanol. Absorbance at 490 nm was measured. Percent viability of cells was calculated by comparison to that of untreated control cells.

#### 2.11.3 Hemocompatibilty

To evaluate the hemocompatibility of the conjugate, 1% RBC suspension was used. 100°μl of the blood suspension was mixed with 100 μl of the conjugate in a U- or V-shaped microtiter plate. After 24 h of incubation, the settling patterns of single and agglutinated red blood cells were observed with the help of a hand lens.

#### 2.11.4 Serum Bactericidal Assay

To 250 μl of treated/non-treated PAO1 cells (10^8^ cells/ml), 500 μl of pre-warmed serum was added and incubated at 37°C. The samples were taken out at 0, 1, 2, and 3 °h post incubation. Different dilutions were prepared and plated on MacConkey’s agar plates and incubated at 37°C to obtain the counts. The results were expressed as follows:

(1) Completely serum-resistant: Organism surviving for 3 h in serum without showing any increase or decrease in viable count after 1 h.
(2) Delayed serum-sensitive: Organism showing significant decrease in cell count after surviving for 1 h.
(3) Promptly sensitive: No viable cells detected after 1 h.

#### 2.12 Statistical Analysis

All the experiments were conducted in triplicate, and results were expressed as means ± standard deviation of different measurements. Significance of data was evaluated with one-way*/*two-way analysis of variance (ANOVA) test using GraphPad Prism version 5.0. The p-value *<*0.05 was considered statistically significant (p-values: * <0.05; ** <0.01; *** <0.001).

## 3 Results and Discussion

### 3.1 Molecular Docking Studies

To clear our perplexities of using catechol as a carrier for zingerone penetration through the outer membrane, a molecular docking study was performed using surface receptor (5FP2) with a novel catechol–zingerone conjugate (**1**) and catechol itself as the natural reference ligand. The ligand poses, docking scores, and involvement of active amino acid residues along with their bond distance for each and respective complexes are manifested in Tables 1, 2. Figure 1 shows 3D cartoon representation of conjugate (**1**) with 5FP2 receptor.

**TABLE 1:** Docking scores (kcal/mol) of conjugate (**1**) and respective natural ligand with Pir A, LasR, PqsR, TraR, and RhlR receptors.

Compounds	Pir A (5FP2)		LasR (2UVO)		PqsR (4JVI)		TraR (IHOM)		RhlR (HM)	
	Ligand pose	D score	Ligand pose	D score	Ligand pose	D score	Ligand pose	D score	Ligand pose	D score
Conjugate **1**	1	−10.78	3	−78.59	5	−20.62	2	−58.83	2	−21.55
Natural ligand	2	Catechol −1.13 Å	2	3-Oxo-C12-HSL −50.129 Å	3	PQS −46.37 Å	3	3-Oxo-C8-HSL −40.96 Å	3	C4-HSL −31.58 Å

**TABLE 2:** Binding interactions of conjugate **1** with various receptors.

PDB ID	Forces involved in interaction with active amino acid residues		
	Hydrogen bond	Hydrophobic interaction	van der Waal’s forces
5FP2	Ser 101A 2.501 Å; Arg 309A 2.061 Å	Leu 92A 2.534 Å; Pro 99A 3.030 Å; Ser 351A 3.877 Å; Glu 353A 3.393 Å	Glu 371A 2.740 Å; Arg 309A 3.001 Å; Pro 99A 2.901 Å
2UVO	—	Lys 42E 3.094 Å; Leu 125G 3.621 Å; Gln 45G 3.132 Å; Asp 43G 3.812 Å	Arg 122E 2.872 Å; Pro 41G 3.060 Å; Lys 42G 2.420 Å; Gly 123G 2.515 Å
4JVI	—	Leu 208A 3.137 Å; Arg 209A 4.423 Å; Val 211A 4.082 Å; Ile 336A 3.853 Å	Leu 208A 2.639 Å; Arg 209A 2.843 Å; Val 211A 2.824 Å; Met 224A 2.884 Å
1HOM	His156B 2.11 Å	Ala 13A 3.049 Å; Ala 121B 2.676 Å; Arg 230B 4.152 Å; Lys 232B 3.227 Å; Ser 160B 3.780 Å	Ala 13A 2.617 Å; Arg 183A 3.099 Å; Ala 121B 2.652 Å; Arg 230 B 3.122 Å; Ser 160B 2.435 Å
HM	Ser142C 2.278 Å	Ser 141C 2.546 Å; Val 92C 3.049 Å; Leu 35C 4.733 Å; Gly 36C 3.331 Å	Leu 35C 2.825 Å; Gly 36C 2.602 Å; Val 92C 2.594 Å; Ser 141C 2.527 Å; Arg 149C 2.886 Å

**FIGURE 1:** Conjugate **1** binding with the 5FP2 receptor.

The selected ligands, conjugate (**1**) and catechol, showed binding affinity toward the receptor indicated by D-score −10.78 and −1.13 Å, respectively. Conjugate (**1**) showed a nine-fold binding affinity toward 5FP2 in comparison to its natural ligand (catechol **1**), with D-score −1.13 Å. This can be attributed to the stearic factor that is helping the conjugate to extend deep into the binding cavity *via* the formation of hydrogen bonding with amino acids Ser 101A and Arg 309A at a bond distance of 2.501 and 2.061 Å, respectively. Furthermore, conjugate (**1**) was found to be engaged with hydrophobic interactions with Leu 92A (2.534 Å), Pro 99A (3.030 Å), Ser 351A (3.877 Å), and Glu 353A (3.393 Å) and van der Waals forces with amino acids Glu 371A, Arg 309A, and Pro 99A by affording bond distance of 2.740, 3.001, and 2.901 Å (Figure 1).

In addition, quorum sensing is a density-dependent cell-to-cell communication adopted by many bacteria by producing diffusible signal molecules, that is, autoinducers (3-oxo-C12-HSL, 3-oxo-C8-HSL, C4-HSL, and PQS) that regulate phenotypic expression of virulence factors and biofilm formation. Further research findings have clearly indicated the role of LasR (PDB: 2UV0), PqsR (4JVI), TraR (1HOM), and the RhlR HM (P54292) system in quorum sensing. Herein, efforts have also been made to understand the binding potential and molecular insights of hypothetically designed catechol–zingerone conjugate toward the enlisted proteins, before carrying out its synthesis. Natural inhibitors (3-oxo-C12-HSL, PQS, 3Oxo 8, and C4 HSL) of all the enlisted proteins from our previously published study were also taken as a reference molecule (Bose et al., 2020).

Good binding affinity has been indicated by conjugate (**1**) toward all the receptors by affording D-score ranging from −20.62 Å to −78.59 Å. Docking studies revealed (Table 1) that further conjugate (**1**) was found to interact in a better way with 2UV0 (−78.59 kcal/mol) and 1HOM (−58.83 kcal/mol) in comparison to reference molecules (3-oxo-C12-HSL and 3-oxo-C8-HSL). This can be associated with well accommodation of the conjugate (1) inside the binding cavity of 2UV0 and 1HOM and highlighting the importance of conjugation and steric factor in quorum quenching potential.

Detailed analysis of the best complex (conjugate **1**: LasR) from Figure 2 indicated hydrophobic interactions of Lys 42E (3.094 Å), Leu 125G (3.621 Å), Gln 45G (3.132 Å), and Asp 43G (3.812 Å) along with van der Waals forces with Arg 122E, Pro 41G, Lys 42G, and Gly 123G at bond distance of 2.872, 3.060, 2.420, and 2.515 Å, respectively, whereas comparable affinity of conjugate 1 was observed for rest of the enzymes is cited in Table 1.

**FIGURE 2:** Conjugate **1** binding with the 2UV0 receptor.

The observations derived from the docking studies revealed its potential to bind with enlisted proteins and can be developed as a promising quorum quenching agent. Furthermore, to support the molecular mechanism, detailed molecular simulation and *in vitro* studies are required.

### 3.2 Design and Synthesis

Natural products are known to treat biofilm-driven infectious diseases worldwide and therefore are gaining attention as alternative therapeutics (Ndjonka et al., 2013). Zingerone is one of the herbal bioactives of dry ginger root which is known to attenuate cell surface properties, making *P. aeruginosa* highly susceptible to killing and innate immunity (Kumar et al., 2014). The present study aimed to exploit iron acquisition pathways for the targeted delivery of zingerone through Trojan horse mechanism to overcome poor bioavailability and limited solubility of drug. To attain this Holy Grail, catechol was synthetically linked to zingerone moiety through a non-hydrolyzable triazole linker. Catechol, a simplified entity with no bulky side groups, is known to use iron uptake systems (Pir & Pfu), therefore mimicking the complex natural siderophores of *P. aeruginosa*.

Furthermore, the selection of zingerone as a drug has an advantage over conventional antibiotics in terms of 1) strong anti-virulent property against Gram-negative organisms due to hydrophobic nature, 2) possess periplasmic target in Gram-negative bacteria, 3) biddable to synthetic modifications without affecting anti-virulent properties, and 4) decreased selection pressure responsible for resistance. Indeed, many examples of pyochelin–antibiotic and pyoverdin–antibiotic conjugates with several types of linkers are reported in the literature (Kinzel et al., 1998; Rivault et al., 2007; Noel et al., 2011; Paulen et al., 2017). However, very few examples of catechol–antibiotic conjugates with non-hydrolyzable linkers are reported in literature (Paulen et al., 2015). The present study divulged the catechol-mediated drug design strategies using herbal bioactive in place of antibiotics as the drug using triazole as a linker.

The stepwise synthesis of the catechol–zingerone conjugate (**1**) has been performed with complete characterization by ^1^H NMR, ^13^C NMR, and mass spectral analysis. The pentafluorophenyl ester (**2**) was synthesized according to previously published protocol in good overall yield of 80% (Baco et al., 2014). The synthesized pentafluorophenyl ester (**2**) and azido propylamine (**3**) (Scheme 2) were reacted, leading to the azido derivative of catechol moiety (**4**) in 80% yield with a molecular mass of 400.13 as identified by mass spectral analysis, and a characteristic IR peak at 2,100 cm^−1^ confirms the azide group as shown in Scheme 1 (Supplementary Figures S1–S4). 3-methoxy-4-(2-propyne-1-yloxy)-phenyl-2-butanone (**6**) was synthesized by nucleophilic substitution reaction of propargyl bromide on zingerone in the presence of potassium carbonate as a base and was formed in quantitative yield showing the characteristic peaks at δ4.7 and δ2.4 in ^1^H NMR and C-C alkyne stretch at 2,125.10 cm^−1^ in FT-IR spectral analysis (Supplementary Figures S5–S7). The azido moiety of catechol (**4**) was then coupled with the acetylene derivative of zingerone (**6**) as shown in Scheme 3 leading to the synthesis of target conjugate (**1**). The prominent peak observed at δ8.2 confirmed the triazole group in conjugate (**1**), which was further subjected to deprotection using methanolic solution of HCl undergoing cleavage of diphenyl dioxole groups, leading to the free functional hydroxyl groups. The final conjugate was purified by column chromatography using CH_2_Cl_2_: methanol (5%).The disappearance of peaks in the aromatic region in ^1^H NMR spectra confirmed the release of diphenyl groups (Supplementary Figures S8, S9). The final synthesis of target conjugate (**1**) was further confirmed by mass spectral analysis (m/z 468.30), FT-IR spectral analysis (Supplementary Figures S10, S11), and elemental analysis (Supplementary Figure S12). Compound was >95% pure as confirmed by HPLC analysis (Supplementary Figure S13).

**SCHEME 2:** Synthesis of compound **2** and compound **3**.

**SCHEME 1:** Synthesis of compound **4**.

**SCHEME 3:** Synthesis of catechol–zingerone conjugate **1**.

### 3.3 Iron Chelation Activity

The iron chelation potential of conjugate (**1**) and the parent drug zingerone and compound 6 was scrutinized on CAS agar plates. Orange halo around the well containing catechol–zingerone conjugate represents the positive reaction, indicating iron binding affinity of the conjugate (**1**) (Figure 3A). The results showed that catechol–zingerone conjugate (**1**), a siderophore mimic, showed iron chelation activity similar to pyochelin, a natural siderophore of *P. aeruginosa*, despite structural modifications. These results are in consensus with the *in silico* results validating strong interactions of the conjugate with outer membrane receptors that is, PirA. Prior literature has also documented that the siderophore component in a conjugate does not necessarily have to be identically a replicate of the natural siderophore (Lin et al., 2019).

**FIGURE 3:** **(A)** Iron chelation potential. **(B)** Antibacterial activity against *P. aeruginosa*. **(C)** Anti quorum activity of synthetic catechol–zingerone conjugate (**1**), compound **6**, and zingerone alone.

### 3.4 Antimicrobial Activity

The antibacterial activity was carried out in Mueller Hinton agar. No activity was observed against *P. aeruginosa* with both conjugate (**1**) and parent drug zingerone (Figure 3B)*.* The results were found to be in agreement with biological activity of pyochelin–zingerone conjugate as stated in previous studies depicting no antibacterial activity (Nosran et al., 2021).

### 3.5 Quorum Quenching Potential

To decrease the selection pressure of antibiotics on bacteria, disarming the pathogen of its virulence instead of killing seems a more promising approach. Since virulence of *P. aeruginosa* is regulated by the quorum sensing systems; therefore, anti-quorum sensing activity of the conjugate at same molar ratios, that is, 50 μM corresponding to sub-MIC of parent drug zingerone was checked using Agrobacterium tumefaciens as the biosensor strain. The colorless halo around the wells containing conjugate as well as parent drug was observed indicating quorum sensing inhibition (Figure 3C). Maximum quorum quenching potential was observed in conjugate (**1**) with zone diameter of 15 mm (Table 3). As per the previous data available in literature, zingerone is a potent inhibitor of ligand–receptor interaction of QS pathways (Kumar et al., 2015), but solubility problem limits its potential as therapeutics (Sharma et al., 2020). Therefore, the possible reason for enhanced quorum quenching potential of conjugate (**1**) observed in the present study might be due to the increased stability as well as solubility of hydrophobic parent drug zingerone after conjugation with catechol moiety through triazole linker.

**TABLE 3:** QSI activity of different compounds against *Pseudomonas aeruginosa* PAO1.

S.No.	Compound	Zone diameter (ZOT)
1	Conjugate **1**	15 mm × 15 mm
2	Compound **6**	8 mm × 8 mm
3	Zingerone	10 mm × 10 mm

### 3.6 Phenotypic Expression of Virulence Factors

For completely hijacking the *P. aeruginosa,* the trail of QS regulated extracellular virulence factors required for the succession of adhesion, colonization and invasion to host cell, needs to be halted (Lau et al., 2004). Since these QS-regulated virulence factors hamper multitudinous cellular functions, therefore potential of the conjugate along with its parent drug was explored for the phenotypic expression of virulence factors. It was observed that the production of all the virulence factors was significantly reduced in the presence of Conjugate (**1**) as well as parent drug, but maximum reduction was showed by siderophore mimic (Table 4). Pyocyanin is a pivotal virulence factor which not only promotes eDNA release in *P. aeruginosa via* hydrogen peroxide production but also intercalates with nitrogenous bases of DNA and creates structural perturbation on double helix structure (Das et al., 2016). There was 45% reduction in pyocyanin production with zingerone alone, which was increased to 57% in the presence of conjugate (**1**) (Figure 4A). Protease and elastase, hydrolytic enzymes degrading the host proteins, reduced more significantly 72% and 60%, respectively, in the presence of conjugate (**1**) than in parent drug (**5**) (Figures 4B,C). Reduction in production of these two enzymes was observed with zingerone alone (Kumar et al., 2015), but no reports are available with siderophore mimics. Pyochelin, an iron chelating siderophore, is another vital virulence factor regulated by the Las system of QS ( Lee et al., 2013). It is known to be associated with sustained inflammatory responses identified in chronic infections (Cornelis and Dingemans, 2013). Upto 40% of pyochelin production was inhibited in the presence of Conjugate (**1**) (Figure 4E). Similarly, the significant reduction in cell-free hemolysin (37%) as well as cell bound hemolysin (77%) was observed (Figures 4F,G). Hemolysins produced by *P. aeruginosa* are known to lyse the RBCs for acquiring iron affecting the host innate response (Gupta et al., 2013). Since alginate is the major polysaccharide present in the extracellular polysaccharide matrix, therefore the effect of conjugate (**1**) was evaluated on alginate production. In addition, alginate helps in attachment of *P. aeruginosa* on surfaces by enhancing cell surface hydrophobicity (Nivens et al., 2001). Highly significant reduction of 50% in alginate production was observed with conjugate **1,** which was furthermore validated by the decreased cell surface hydrophobicity indicating declined colonization to host surfaces (Figures 4D,H). Prominent downturn in production of QS-regulated virulence factors in the presence of conjugate (**1**) might be due to the increased membrane permeability through the iron acquisition pathway, thereby clogging the QS network.

**TABLE 4:** Phenotypic expression of virulence factors in the presence and absence of conjugate **1**, compound **6**, and Zingerone **5**.

Compound	Pyocyanin (µg/ml)	Protease (U/l)	Elastase (U/l)	Alginate (OD_500_)	Pyochelin (OD_510_)	Cell-free hemolysin (mg/ml)	Cell-bound hemolysin (mg/ml)	Cell surface hydrophobicity (%)
Control	3.132	0.545	1.225	0.618	0.132	3.000	4.900	75
Conjugate **1**	1.360	0.155	0.497	0.308	0.080	1.900	1.099	35
Compound**6**	1.680	0.230	0.640	0.400	0.104	2.800	2.500	60
Zingerone **5**	1.700	0.240	0.655	0.411	0.090	2.000	1.200	45

**FIGURE 4:** Effect of sub-MIC of catechol–zingerone conjugate (**1**), compound (**6**), and zingerone alone, on the virulence factors in *P. aeruginosa*. **(A)** Pyocyanin, **(B)** protease, **(C)** elastase, **(D)** alginate, **(E)** pyochelin, **(F)** cell-free Hemolysin, **(G)** cell-bound hemolysin, and **(H)** cell surface hydrophobicity.

### 3.7 Curtailment of Motility Phenotypes

QS-related motility phenotype in *P. aeruginosa* acts as one of the vital virulence determinant due to its role in colonization to establish biofilms (Taguchi et al., 2010). In order to investigate the impact of siderophore mimic that is, catechol–zingerone conjugate on the motility phenotypes (swimming, swarming, and twitching), conjugate (**1**) along with the parent drug zingerone was evaluated on swim, swarm, and twitch plates *in vitro*. In the present study, swarming, swimming, and twitching motilities of *P. aeruginosa* in the presence of 50 μΜ catechol–zingerone conjugate (**1**) were reduced significantly as found with the parent drug, indicating non-interference of catechol moiety with antimotility activity of zingerone (Figures 5A–C). However, the antimotility effect of pyochelin–zingerone conjugate as stated in the previous study depicted moderate antimotility effect against *P. aeruginosa,* which might be due to the bulky side groups of pyochelin (Kumar et al., 2015; Nosran et al., 2021). The results of the present study were in agreement with those of the previous studies where a reduction in swimming, swarming, and twitching motility of *P. aeruginosa* was observed at sub-MIC of zingerone (Kumar et al., 2015). Since motility phenotypes are involved in biofilm formation; therefore, it can be hypothesized that Trojan horse drugs inhibiting motility can be the probable candidates for inhibition of biofilm formation by *P. aeruginosa* and hence can be considered for development of therapeutics.

**FIGURE 5:** Antimotility effects of catechol–zingerone conjugate (**1**), compound (**6**), and zingerone alone. Swarming **(A)**, swimming **(B)**, and twitching **(C)** motility patterns of *P. aeruginosa* in absence (control) and presence (tests) of sub-MIC of catechol–zing conjugate **1**, compound **6**, and zingerone alone.

### 3.8 Devitalization of Biofilm of *Pseudomonas aeruginosa*

The biofilm-forming ability of *P. aeruginosa* is the prime partner in crime as it involves multiple bacterial machinery. Importantly, past studies have shown an indirect link between biofilm formation and QS through the control of motility phenotypes as well as alginate production (Rasamiravaka et al., 2015). The antibiofilm activity of zingerone alone has previously been reported against *P. aeruginosa* where phyto-molecule mimics the signal molecules (Kumar et al., 2015). The biofilm-forming capacity of *P. aeruginosa* in the presence of conjugate (**1**) as well as parent drug was evaluated qualitatively. In the presence of conjugate (**1**), *P. aeruginosa* showed weak adherence as compared to control which showed strong adherence to polypropylene tubes (Figure 6). Furthermore, the effect of the conjugate on different stages of biofilm formation (young, peak, and old) of *P. aeruginosa* was studied up to 7 days. Results inferred that biofilm formation was inhibited in the presence of conjugate (**1**) as well as parent drugs (Figure 7A). However, the maximum inhibition was observed in the presence of conjugate (**1**), which might be due to enhanced cell penetration of zingerone through extracellular polymeric substances and stability of zingerone when conjugated to catechol, a xenosiderophore. A significant reduction in peak-day biofilm was observed in all the regimes, but maximum reduction was observed in conjugate indicating anti-biofilm activity (Figure 7B **)**. EPS, being the vital functional component of *P. aeruginosa* biofilm matrix, was quantified in the presence and absence of conjugate as well as parent drugs. Treatment with conjugate significantly deteriorated the EPS production, resulting in devitalization of biofilm matrix (Figure 7C). To explore the ability of conjugate to eliminate pre-formed peak-day biofilm, biofilm eradication was performed. Enhanced anti-biofilm effect of the conjugate might be due to targeted delivery of zingerone through iron acquisition pathways as shown by *in silico* analysis.

**FIGURE 6:** Qualitative biofilm formation by *P. aeruginosa*. **(A)** Untreated control, **(B)** catechol–zingerone conjugate (**1**), **(C)** compound (**6**), and **(D)** zingerone alone. Strong adherence (+++), moderate adherence (++), and weak adherence (+).

**FIGURE 7:** **(A)** Inhibition pattern of *P. aeruginosa* biofilms (young, peak, and old), **(B)** percentage biofilm eradication as quantified by crystal violet assay, and **(C)** percentage EPS estimation of the biofilm matrix by using the Congo red binding assay in absence and the presence of sub-MIC of catechol–zingerone conjugate (**1**), Compound (**6**), and zingerone alone.

The antibiofilm effect of the conjugate was further confirmed by the light microscopy and FE-SEM analysis. Thinner and delicate biofilms with loose adherence were observed under light microscope in the presence of conjugate (**1**), which is indicative of reduced biofilm as compared to control (Figures 8A,B). Furthermore, conjugate treatment distorted the cell surface, leading to the leakage of cell materials as evidenced from FE-SEM micrographs (Figures 8C,D).

**FIGURE 8:** Microscopic visualization of *P. aeruginosa* biofilms. Peak-day biofilm formed in the absence **(A,C)** and presence **(B,D)** of sub-MIC of catechol–zingerone conjugate **1** by light microscopy at ×100 **(A,B)** and scanning electron microscopy **(C,D)**.

### 3.9 Unfurling the Mode of Action

Mode of action of the catechol–zingerone conjugate (**1**) might be attributed to its ability to penetrate or disrupt the bacterial plasma membrane. To understand the underlying mechanism, crystal violet uptake assay was performed. The results suggested that treatment with the 100 μΜ catechol–zingerone conjugate (**1**) enhanced membrane permeability of *P. aeruginosa* (Figure 9A). Furthermore, release of cellular contents followed by SDS-PAGE was investigated to confirm the increased membrane permeability. Present results inferred that treatment of *P. aeruginosa* with catechol–zingerone conjugate 1 led to the release of intracellular contents represented as separate bands on SDS-PAGE (Figures 9B,C). This might be due to the competitive binding of catechol zingerone conjugate (**1**) in the binding pocket of Las and Rhl receptor, thereby seizing the pathogen of its virulence by downregulating lasI and rhlI genes as shown by *in silico* studies. These results were found to be in agreement with the action of thymol as stated in previous study, depicting increased membrane permeability and release of cellular contents in the presence of thymol (Chauhan and Kang, 2014). However, not much information regarding conjugate is available.

**FIGURE 9:** **(A)** Crystal violet uptake of catechol–zing conjugate (**1**). **(B)** Effects of catechol–zing conjugate on release of cellular materials on *P. aeruginosa* based on absorbance recorded at 260 nm. **(C)** Time-dependent proteins released into the supernatant, detected by using SDS-PAGE.

### 3.10 *Ex Vivo* Efficacy

Since innate immune defense provided by the serum and macrophages forms the first line of defense against invading pathogens. Therefore, it becomes imperative to evaluate the effect of conjugate on *ex vivo* efficacy of catechol–zingerone conjugate (**1**) in terms of hemocompatibility, cell cytotoxicity, and serum susceptibility. For the contemplation of the conjugate as a new treatment regime, hemocompatibility testing was performed. Results reflected that incubation of RBCs with conjugate (**1**) in round-bottom 96-well plate resulted in button formation, indicating hemostability as compared to the control with cell lysis (Figure 10A). Cytotoxicity analysis of activated peritoneal macrophages treated with the conjugate was performed through MTT. Formation of formazen crystal in the presence of conjugate accorded the cell viability, indicating safety of the conjugates (Figure 10B). Activated macrophages producing formazen crystal indicates cell viability (Mosmann, 1983). Furthermore, serum susceptibility assays demonstrated the significant decrease in log count within 30 min of the treatment followed by complete evacuation within 2 h as compared to control showing serum resistance (Figure 10C). Conversion of delayed serum-susceptible PAO1 cells to prompt serum susceptibility in the presence of conjugate might be due to the surface alterations.

**FIGURE 10:** Influence of catechol–zingerone conjugate **1** treatment on **(A)** Hemocompatibility, **(B)** cell cytotoxicity, and **(C)** serum susceptibility against *P. aeruginosa*.

## 4 Conclusion

This work illustrates that conjugation of natural bioactive, that is, zingerone with catechol, a xenosiderophore of *P. aeruginosa*, using click triazole as a linker can act as a novel Trojan horse conjugate. This hybrid drug was designed for targeted drug delivery exploiting the bacterial iron acquisition pathway. Docking studies suggested that conjugate (**1**) can interact with membrane receptor PirA and the quorum sensing signal receptors with low binding affinity, indicating less or no steric hindrance of catechol moiety on drug components. This conjugate (**1**) was synthesized using a non-hydrolyzable linker which showed iron chelation activity. Furthermore, conjugate (**1**) can inhibit QS-activity, reduce virulence factor production, and disrupt biofilm formation, which is crucial for pathogenesis of *P. aeruginosa.* This study proves that conjugate (**1**) has the potential of modulating the surface properties of *P. aeruginosa,* leading to its enhanced serum susceptibility with no cell cytotoxicity. To the best of our knowledge, this is the first report to investigate the potential of catechol zingerone conjugate (**1**) in attenuation of virulence factors and biofilm formation in *P. aeruginosa*. However, more detailed *in vivo* studies are required to make use of conjugate (**1**) in clinical practice.

## Data Availability

The original contributions presented in the study are included in the article/Supplementary Material; further inquiries can be directed to the corresponding authors.

## Abbreviations

AMR, antimicrobial resistance; DMSO, dimethyl sulfoxide; EPS, exopolysaccharide; FE-SEM, field emission scanning electron microscopy; FT-IR, Fourier transform infrared; HSL, homoserine lactone; MDR, multidrug resistance; MS, mass spectroscopy; NMR, nuclear magnetic resonance; PAO1, *Pseudomonas aeruginosa*; QS, quorum sensing; SDS-PAGE, sodium dodecyl sulfate–polyacrylamide gel electrophoresis.
